# Structural and Functional Properties of Activator Protein-1 in Cancer and Inflammation

**DOI:** 10.1155/2022/9797929

**Published:** 2022-05-26

**Authors:** Pritam Bhagwan Bhosale, Hun Hwan Kim, Abuyaseer Abusaliya, Preethi Vetrivel, Sang Eun Ha, Min Yeong Park, Ho Jeong Lee, Gon Sup Kim

**Affiliations:** ^1^Research Institute of Life Science and College of Veterinary Medicine, Gyeongsang National University, Gazwa, Jinju 52828, Republic of Korea; ^2^Biological Resources Research Group, Gyeongnam Department of Environmental Toxicology and Chemistry, Korea Institute of Toxicology, 17 Jegok-gil, Jinju 52834, Republic of Korea

## Abstract

The transcriptional machinery is composed of numerous factors that help to regulate gene expression in cells. The function and the fundamental role of transcription factors in different human diseases and cancer have been extensively researched. Activator protein-1 (AP-1) is an inducible transcription factor that consists of a diverse group of members including Jun, Fos, Maf, and ATF. AP-1 involves a number of processes such as proliferation, migration, and survival in cells. Dysfunctional AP-1 activity is seen in several diseases, especially cancer and inflammatory disorders. The AP-1 proteins are controlled by mitogen-activated protein kinases (MAPKs) and the NF-*κ*B pathway. AP-1 inhibitors can be actively pursued as drug discovery targets in cancer therapy when used as a treatment to halt tumor progression. The consumption of phytochemicals in the diet is related to decreasing the incidence of cancer and proves to exhibit anticancer properties. Natural product targets AP-1 are effective cancer prevention and treatment options for various cancer types. Targeting AP-1 with natural products is an effective cancer treatment option for different cancer types. This review summarizes AP-1 subunit proteins, their structures, AP-1-related signaling, and its modulation by natural bioactive compounds.

## 1. Introduction

Activator protein-1 (AP-1) is a transcription factor comprising heterodimeric complexes and involves in a broad range of biological activities such as cell differentiation, survival, apoptosis, proliferation, cell transformation, and migration [1]. It was one of the earliest transcription factors (TFs) discovered in mammals. The TFs are the proteins that regulate gene expression by changes in mRNA levels, which further leads to necessary biological changes [2]. Identifying the molecular processes is an essential step to understanding the etiology and underlying causes of diseases. AP-1 has received a lot of attention as a therapeutic drug development target in recent years, and it has been identified as a substantial and influential target for several human disorders [3]. The AP-1 complex has been related to the onset and progression of inflammatory diseases, cancer, asthma, rheumatoid arthritis, and psoriasis. It is a predominant target for various diseases including cancer and inflammation [4]. Previously, AP-1 is believed to be oncogenic; however, current studies have changed this perception as some AP-1 proteins have been shown to have tumor-suppressive activity. So, AP-1 has double-edged action that may be anti-oncogenic by promoting apoptosis and oncogenic by encouraging cell survival [5].

The literature reviewed by *James E*. *Darnell* has summarized a list of hyperactive TFs found in numerous cancer cells that are considered potential targets for anticancer drug development [6]. Altered TF activity is an important factor in various cancer types, generally triggered by several direct modes, including gene duplication, chromosomal translocations, point mutations, and variable expression levels [6, 7]. In addition, indirect mechanisms may affect TF binding to the target DNAs via noncoding DNA mutations in the promoter region. TFs implicated in disease progression can be potential targets to block EMT, increased differentiation, replicative immortality, and immune invasion [8]. It is reported that TFs link with epigenetic modifiers to control the gene expressions responsible for the cellular oncogenic phenotype. A thorough understanding of TFs and epigenome functioning during disease development will offer prospects to design novel drugs [9]. One such area is the rise of AP-1 inhibitors, particularly for inflammatory diseases and cancer. There is a great scope to design and develop AP-1 inhibitors for therapeutic agents in disease treatment [3, 10]. In the current work, we attempt to provide an overview of the AP-1 family, its functions, and its associated signaling pathways.

## 2. Structure of AP-1 Proteins and Their Types

AP-1 comprises a homo- and heterodimeric complex formed by proteins from the basic-region leucine zipper (bZIP), such as Jun, Fos, Maf, and ATF. The AP-1 transcription factor is formed by the dimerization of a characteristic bZIP domain (basic-region leucine zipper) in the Fos and Jun subunits. The AP-1 interacting proteins and their subfamilies are summarized in Table 1. The bZIP domains recognize various response elements (REs) in genomic regions, and they are necessary for DNA binding and dimerization with AP-1 [11]. The leucine zipper is a structural motif that forms an extended *α*-helix with leucine as the seventh amino acid [12]. The AP-1 family comprises multiple proteins that are expressed in cells in a stage-dependent fashion in development and regulate the transcription of genes at various levels. The structure of AP-1 is shown in Figure 1 PDB code 1Fos [13].

## 3. Interaction among AP-1 Family Subunits

The AP-1 family of transcription factors comprises heterodimers and homodimers of Jun, Fos, ATF, and MAF. The proto-oncogenes c-Jun and c-Fos were the first to be discovered and extensively documented as AP-1 components. Jun was discovered in the genome of transformed cells of an avian sarcoma virus 17 with a replication defect (ASV17). Jun proteins are highly conserved in terms of amino acid sequence and structure, with 75% amino acid homology in the DNA-binding domain and leucine zipper regions [14]. Jun proteins form both homo- and heterodimeric complexes in their gene members. Following the identification of v-Jun proteins, the C-terminal region was found to be similar to the DNA-binding domain of yeast TF named GCN4 [15, 16]. Using this particular piece of DNA for affinity chromatography, the mammalian c-Jun was co-purified with c-Fos, establishing that the first AP-1 forms heterodimer with c-Fos and c-Jun. Jun-Jun and Jun-Fos dimers preferentially bind to the phorbol 12-O-tetradecanoate-13-acetate (TPA)-responsive element (TRE; Consensus DNA sequence TGACTCA) [17]. AP-1 subunit members possess distinct dimerization capability [18], whereas c-Maf and Nrl can form heterodimers with c-Jun and c-Fos and Maf-related proteins, such as MafB, MafF, MafG, and MafK, form dimers only with Fos but not Jun. Certain dimers have a weak affinity for DNA sequences that deviate from the consensus AP-1 protein and can form unique DNA binding and TF activity interacting with other proteins outside [19].

The Fos oncogene was first reported in two retroviruses, namely Finkel-Biskis-Jinkins murine osteosarcoma virus (FBJ-MSV) and the Finkel-Biskis-Reilly murine osteosarcoma virus (FBR-MSV) [20]. The Fos gene subunits of TFs include c-Fos (the human homolog of the retroviral oncogene v-Fos), FosB, Fra1, and Fra2, and smaller FosB [14]. Unlike the Jun proteins, however, c-Fos and other members of the Fos preferentially form heterodimers (and not homodimers) to transcriptionally activate AP-1 containing promoter constructs in the cells [21]. Splicing variant of FosB, i.e., ΔFosB, follows a different mode of regulation. Some drug treatments show gradual induction of ΔFosB; however, it persists for very long periods. A recent study proposed that ΔFosB is a molecular link between acute drug effects and the long-term neural and plastic adaptations that lead to addiction [22]. Fra-2 is another Fos member identified as a 46 kDa protein in fibroblasts of a chicken embryo that possesses high homology with FosB and Fra-1 [23]. Some cancer cell lines express a higher level of Fra-2 compared with noncancerous ones. Fra-2 is involved in several cellular and physiological activities, for example, spermatogenesis, keratinization, cell differentiation, and cornification of the skin epithelium [24]. Fra-2 also can be a specific novel drug target in lupus nephritis [25].

Maf was reported first in the genome of an avian transforming retrovirus, AS42 [26]. The Maf units are classified into two subgroups based on their molecular size: small Maf TFs (150–160 amino acids: MafF, MafG, and MafK) and large Maf TFs (240–340 amino acids: MafA, MafB, c-Maf, and Nrl) [27]. Loss of function of small Maf TFs results in various disease phenotypes, for example, progressive cataracts, neuronal degeneration, embryonic lethality, and thrombocytopenia [28]. c-Maf is overexpressed in multiple myeloma, which improves tumor-stroma interaction, required for macrophage self-renewal [29]. By regulating c-Maf, duct cells in the pancreas turned into insulin-secreting cells, for the treatment of diabetes mellitus [30]. Jun-ATF dimers or ATF homodimers prefer to bind to the cAMP-responsive element (CRE; DNA sequence TGACGTCA). ATF complexes bind to either heptameric or octameric AP-1-binding sites and are mediated differentially by cellular signaling pathways and oncogene products [31]. Dimerization partners are shown in Table 2.

## 4. Role of AP-1 in Signaling Pathways

### 4.1. NF-*κ*B Pathway

Nuclear factor-*κ*B (NF-*κ*B) is a class of inducible TFs, which regulates a diverse set of genes involved in inflammatory and immune responses [32]. AP-1 and NF-*κ*B regulate critical processes such as embryonic development, lymphoid differentiation, inflammation, apoptosis, and oncogenesis [33]. Various physiological and environmental stimuli promote NF-*κ*B and AP-1 activity [34]. I*κ*B, an inhibitor of NF-*κ*B, controls its activity by forming an NF-*κ*B and I*κ*B complex in the cytoplasm [35]. In response to diverse stimuli, I*κ*B kinase complex (IKK) phosphorylates the I*κ*B bound to the NF-*κ*B complexes as substrates [36]. Even NF-*κ*B and AP-1TFs are regulated by distant mechanisms, they are activated by a similar set of stimuli [37]. JNK is activated through stress or inflammatory cytokines subsequently nuclear translocation of the NF-*κ*B and the I*κ*B complexes (Figure 2). Furthermore, there is a potential that NF-*κ*B and AP-1 may affect each other's actions, broadening the scope of these two inducible TFs. The findings show that NF-*κ*B and AP-1 have an important role in regulating FasL in the Fas-mediated thymineless death of colon cancer cells [38]. Therefore, AP-1 and NF-*κ*B can be better targets for cancer prevention [39].

### 4.2. MAPKs Pathway

AP-1 activity is influenced by growth factors, cytokines, polypeptide hormones, neurotransmitters, viral and bacterial infections, and chemical and physical stresses. These stimuli trigger to activate the mitogen-activated protein kinase (MAPK) pathway [40]. These signals lead to the MAPK activation through phosphorylation of serine/threonine residues of target proteins, resulting in the activation of extracellular signal-regulated kinase (ERK), p38 kinase, and c-Jun N-terminal kinase (JNK) [41]. The MAPK pathway forms three- or four-tiered signaling modules in which MAPK has activated a MAPK kinase (MAPKKK). Small G-protein, as Ras, activates the MAPKKK. The MAPKKs (MKK4 and MKK7) activate JNK [42]. MEK1 and MEK2 stimulate ERKs, whereas MKK3 and MKK6 activate p38. Once MAPKs are activated, they modulate downstream TFs that are necessary to induce the transcription of Fos and Jun genes, increasing the expression of the AP-1 complex [3]. TFs cause the induction of Fos, which is then activated by p38, JNKs, and ERKs. The Jun expression is induced by MEF2C, ATF2, and Jun, which is further activated by p38 and JNK phosphorylation (Figure 3). When AP-1 and other cellular factors are activated, they regulate cellular proliferation, change in the gene expression, apoptosis, differentiation, and migration in response to stimuli, for example, growth factors, oncogenic transformation, stress, cytokines, and noxious stimuli [43].

## 5. Functions of AP-1 Associated with Inflammation and Cancer

### 5.1. AP-1 and Inflammation

Inflammation refers to the complex interactions among soluble factors and cells that can occur in any tissue as a result of infectious, traumatic, post-ischemic, autoimmune, or toxic injury [44]. Tremendous progress has been achieved in identifying the molecular and cellular processes associated with inflammatory responses to infection and tissue injury [45]. The inflammatory response is regulated through a diverse set of mediators that create complex regulatory networks, and it is a powerful weapon employed by the innate and adaptive immune systems to maintain the tissue and cell homeostasis [46]. The inflammatory mechanism has a great role in autoimmune diseases and cancer. Improper activation of the immune system happens when inflammatory cells and proteins attack and damage healthy cells, resulting in the overproduction of immune cells leading to inflammatory disorders such as chronic inflammatory diseases, psoriasis, systemic lupus erythematosus, psoriatic arthritis, and rheumatoid arthritis [47]. In these diseases, chemotactic proteins and cytokines are produced, attracting innate and adaptive immune cells and exacerbating the inflammatory response. As AP-1 is activated by environmental and physiological stressors such as UV radiation, cytokines, and infections, which are known to the formation of free radicals, AP-1 also controls MMPs, cytokines, and extracellular matrix components [48]. Reported studies have shown that TFs activation controls through similar intracellular signal pathways. Inflammatory cytokines and stress activate JNK, which usually accompanied NF-*κ*B translocation and other genes essential for AP-1 activation. The MAPK pathway activates JNK and I*κ*B kinase complexes and provides insights into the interaction between AP-1 and NF-*κ*B signaling pathways [33, 49]. AP-1 suppression may be a useful therapeutic approach for treating inflammatory processes as it reduces inflammatory cytokines and chemokines.

Sophoraflavanone M, a flavonoid, inhibits proinflammatory mediators by both JNK/AP-1 and NF-*κ*B signaling pathways in LPS-stimulated macrophages [50]. Apigenin-7-O-*β*-D-glucuronide, a flavonoid isolated from species *Juglans sigillata* fruit husks, has numerous medicinal properties and effectively reduces inflammatory responses in LPS-stimulated RAW 264.7 cells by downregulating inflammatory-related gene expression via suppression of AP-1 and MAPK signaling pathways [51]. Chrysoeriol is a flavonoid with diverse biological properties and reduces COX-2 expression in LPS-stimulated murine macrophages via NF-*κ*B, AP-1, and MAPK regulation by TLR4/MyD88 signaling pathway [52]. Silibinin decreases inflammation induced by silica dioxide nanoparticles with inhibition of TXNIP/MAPK/AP-1 signaling [53]. Anti-inflammatory effects of the various parts of *longan* including flowers, seeds, and pulps inhibit LPS-stimulated nitric oxide production in macrophages by inhibiting NF-*κ*B and AP-1 signaling pathways [54]. Taken altogether, AP-1 can be a therapeutic target for treating underlying inflammatory diseases.

### 5.2. AP-1 and Cancer

Numerous studies demonstrated that AP-1 members play a key role in cancer progression. The c-Jun and c-Fos were discovered as retrovirus-activated genes with oncogenic potential in avian and mammalian cells [14]. The effects of AP-1 on several cancer “hallmarks” demonstrate its pro-oncogenic and anti-oncogenic activities [5]. Although AP-1 proteins are thought to be carcinogenic, current research has discovered that JunB and c-Fos have tumor-suppressing activity, providing insights into the molecular processes that control the oncogenic and anti-oncogenic functions of AP-1 in tumorigenesis [55]. Extrinsic death receptor pathways, such as JNK, Jun/AP-1, and FasL, have been studied for their importance in controlling fibroblast, neuronal cell fate, and lymphoid. JNK is activated by the MAPK cascade, which phosphorylates Jun, resulting in increased transcription of target genes involved in apoptosis. Both FasL and TNF*α*, which encode proapoptotic Jun genes, contain AP-1-binding sites [56]. Increased AP-1 activity found in multiple human cancer cell lines indicates that AP-1 plays a role in tumor growth. *Bernstein and Colburn* were the first to suggest that transformation-resistant JB6 cells failed to activate AP-1 in response to tumor promoters, while AP-1 response was intact in the transformation-sensitive JB6 cells [57]. Thus, AP-1 has a great potential for both cancer prevention and treatment. The molecular mechanisms by which AP-1 activation leads to apoptosis, or survival, remains a formidable challenge and we have only begun to determine the AP-1-regulated target genes that contribute to the apoptotic process [58]. EMT is crucial in not only in tumor invasion and metastasis but also in apoptosis. Several studies have reported contribution of AP-1 to EMT through JunB in malignancies. In some studies, the JunB pathway might be used as a therapeutic target for inhibiting metastasis [59]. AP-1 inhibitors can be used as a therapeutic approach to inhibit tumor progression and invasion [4]. Among the Jun proteins, c-Jun is unique in its ability to positively regulate cell proliferation through the repression of tumor suppressor gene expression and function and induction of cyclin D1 transcription [40]. The activation of the c-Jun and AP-1 complex induces positive regulators of the cell cycle such as cyclin D1. JunB and JunD upregulate tumor suppressor genes and represses cyclin D1 [60]. Fibroblasts from mice overexpressing JunB showed decreased proliferation, whereas JunD-deficient immortalized fibroblasts showed increased proliferation, indicating that JunD could both positively and negatively mediate the cell cycle process [5]. Phytochemicals have the ability to modulate TFs including AP-1.

Apigenin inhibited IL-1*β*-induced expression of the urokinase-type plasminogen activator receptor by reducing MAPK-mediated AP-1 and NF-*κ*B signaling in bladder cancer cells [61]. Nobiletin impaired cell proliferation by AP-1 signaling in mammary carcinogenesis in rats [62]. Fisetin, a flavonol, activates the hippo and JNK/ERK/AP-1 signaling in human osteosarcoma cells, inhibiting proliferation and inducing apoptosis via ZAK overexpression [63]. Orientin treated along with TPA in MCF7 breast carcinoma cells suppresses IL-8 and MMP-9 by PKCα/ ERK/AP-1/STAT3 pathway [64]. Kaempferol causes inactivation of JAK-STAT and NF-κB, and AP-1 in LPS-induced RAW 264.7 macrophage [65]. Significant evidence shows that the expression of AP-1 is linked to several malignancies. The role of AP-1 is explained in Figure 4.

### 5.3. The Role of AP-1 in Cancer: Oncogenic or Anti-Oncogenic?

AP-1 proteins are considered to be oncogenic but have recently been shown to have tumor suppressor activity. Fos and Jun proteins were first identified as the viral oncoproteins. When the cellular counterparts of the viral oncoproteins were discovered, the upregulation of AP-1 proteins by overexpression or by oncogenic RAS was found to correlate with a positive effect on cell transformation [5]. Some Jun and Fos proteins not only lack transforming action but can also inhibit carcinogenesis. While c-Jun is carcinogenic, JunB and JunD exhibit anticarcinogenic properties [55]. According to some research, JunD is a negative regulator of cell growth. The decision of whether AP-1 is oncogenic or anti-oncogenic may be regulated by the antagonistic activity of various Jun proteins, but it is also likely regulated by tumor form, tumor stage, and tumor genetic background [66]. AP-1 acts as a double-edge sword in tumor development as it exhibits both anti-oncogenic and oncogenic effects by regulating cell signaling.

## 6. Conclusion

In conclusion, it is critical to target AP-1 to control diseases like cancer. However, owing to its importance in a wide range of biological activities, it is a promising drug target. Natural bioactive compounds inhibited AP-1, indicating that it may play a potential role in cancer and inflammation (Table 3). Natural products are considered to have lesser side effects than synthetic drugs. AP-1, on the other hand, can act as a double-edged sword in tumor development. Thus, natural products that target AP-1 have the potential to be of significant research interest in cancer prevention and therapy.

## Figures and Tables

**Figure 1:** Structure of activator protein (AP)-1. The carboxy-terminal regions of *α*-helixes align to form parallel “coiled coils”, while the amino-terminal regions make base-specific contacts with DNA in the major groove (PDB code 1Fos). Coils forming leucine zipper in blue and pink are c-Fos and c-Jun, respectively.

**Figure 2:** Illustration of the NF-*κ*B pathway in AP-1. NF-*κ*B is an inducible transcription factor that activates various genes and thereby regulates the inflammatory process.

**Figure 3:** MAPK- and AP-1-related signaling pathways. MAPK signaling integrates signals from diverse stimuli and elicits appropriate responses such as cellular proliferation, development, apoptosis, and inflammatory responses in cells. Schematic representation of MAPK and AP-1 pathways explained in the text.

**Figure 4:** Schematic representation of AP-1 in cancer. AP-1 transcription factor regulates gene expression in response to various stimuli and controls the number of cellular processes in cells.

**Table 1:** List of different AP-1 transcription factor subunits JUN, FOS, MAF, and ATF.

JUN	FOS	MAF	ATF
c-Jun	v-Fos	c-Maf	ATF2
JunB	c-Fos	MafB	LRF1/ATF3
JunD	FosB	MafA	B-ATF
	Fra-1	MafG/F/K	JDP1
	Fra-2	Nrl	JDP2

**Table 2:** AP-1 (activator protein-1) subunits and their binding partners.

Subunits	Binding partners
c-Jun	JunB, JunD, c-Jun, FosB, Fra1, Fra2, ATF2, ATF3, BATF, c-MAF, Maf G/F/K, MafB
c-Fos	c-Jun, JunB, JunD, ATF2, ATF4, c-Maf, MafB, Maf G/F/K
JunB	c-Maf, ATF3
JunD	ATF4
MafB	Fra-1, Fra-2

**Table 3:** Representative examples of natural compounds analyzed for their anti-inflammatory and anticancer properties by altering cellular pathways in different cell lines.

Flavonoid	Source species	Cell line	Targeted pathway	References
Sophoraflavanone M	Sophora flavescens Ait	Murine macrophage RAW264.7	NF-*κ*B and JNK/AP-1	[50]
Naringenin	*Citrus paradisi*	A549	JNK/AP-1	[67]
Quercitrin	*Fagopyrum tataricum*	JB6 P+	AP-1 and MAPK	[68]
Kaempferol	*Smilax china*	RAW 264.7 macrophages	NF-*κ*B, AP-1, and JAK-STAT	[65]
Orientin	*Adonis vernalis*	MCF-7	PKC*α*/ERK/AP-1/STAT3	[64]
Fisetin	*Acacia greggii*	Human osteosarcoma cells	JNK/ERK/AP-1	[63]
Epicatechin	*Acacia catechu* L.f.	Mouse primary astrocytes	Nrf2 and AP-1	[69]
Chrysin	*Passiflora caerulea*	AGS	MMP-9/AP-1/ERK/JNK	[70]
Glabridin	*Glycyrrhiza glabra*	Huh7 and Sk-Hep-1	NF-*κ*B and AP-1	[71]
Acacetin	*Robinia pseudoacacia*	A549	NF-*κ*B and AP-1	[72]

## Data Availability

Data can be obtained with prior permission.
